# MicroRNA‐612 inhibits cervical cancer progression by targeting NOB1

**DOI:** 10.1111/jcmm.14985

**Published:** 2020-01-22

**Authors:** Yang Jin, Xu Zhou, Xiaoxiao Yao, Zhuo Zhang, Manhua Cui, Yang Lin

**Affiliations:** ^1^ Jilin Provincial Key Laboratory on Molecular and Chemical Genetic The Second Hospital of Jilin University Changchun China; ^2^ Department of Obstetrics and Gynecology The Second Hospital of Jilin University Changchun China; ^3^ Department of Orthopedics China‐Japan Union Hospital of Jilin University Changchun China

**Keywords:** cervical cancer, invasion, miR‐612, nin one binding protein, proliferation

## Abstract

Recently, many studies have shown that microRNA (miR)‐612 is involved in cancer progression. However, the role of miR‐612 in cervical cancer remains unclear. The present study aims to investigate the biological effects of miR‐612 on cervical cancer. The expression of miR‐612 in cervical cancer tissues and cell lines was analysed by quantitative reverse transcription‐polymerase chain reaction. The effect of miR‐612 cell proliferation, migration, invasion and apoptosis was studied by appropriate methods. Protein expression was determined by Western blot analyses. Bioinformatics analysis and luciferase reporter assays were performed to clarify the relationship between miR‐612 and nin one binding protein (NOB1). A xenograft model was established to examine the role of miR‐612 in vivo tumorigenesis. Cervical cancer tissues and cell lines showed down‐regulation of miR‐612 expression, which was associated with the Fédération Internationale de Gynécologie et d'Obstétrique (FIGO) stage and lymph node metastasis. Functional assays revealed that miR‐612 overexpression significantly suppressed cervical cancer cell proliferation, migration and invasion in vitro and delayed tumour growth in vivo. Mechanically, miR‐612 targeted NOB1 in cervical cancer cells, revealing a negative correlation between miR‐612 and NOB1in cervical cancer samples. NOB1 overexpression partially reversed the inhibitory effects of miR‐612 overexpression in cervical cancer cells. Taken together, these findings indicate that miR‐612 functions as a tumour suppressor in cervical cancer and suggest that miR‐612 may be a potential target in the therapeutic intervention of this malignancy.

## 1 INTRODUCTION

Cervical cancer is the second most prevalent gynaecological malignancy in women, and its incidence has increased significantly worldwide.^1^ Despite that advanced treatments including surgery, radiotherapy, chemotherapy and combined radio‐chemotherapy have improved the overall survival rate, the prognosis and 5‐year overall survival of patients with locally advanced or metastatic cervical cancer remain poor because of the development of resistance to current clinical treatments.^2^, ^3^ Thus, there is an urgent need to explore the underlying molecular mechanisms of cervical cancer for its diagnosis and treatment.

MicroRNAs (miRNAs) are a class of small (19‐25 nucleotides in length) non‐coding RNA molecules that regulate gene expression by binding to the 3'‐untranslated regions of target mRNA.^4^ Accumulating evidence has suggested that miRNAs exert critical effects on cellular processes such as proliferation, stemness, apoptosis, invasion and metastasis.^5^, ^6^ Moreover, miRNAs reportedly play essential roles as oncogenes or tumour suppressors in the tumorigenesis and progression of various cancers,^7^, ^8^ including cervical cancer.^9^, ^10^ Therefore, miRNAs may become novel therapeutic targets and potential clinical biomarkers for cervical cancer.

MicroRNA‐612 (miR‐612), located on chromosome 11, has recently been reported to be down‐regulated and play a potential role as a putative tumour suppressor in several types of human cancers, including hepatocellular carcinoma,^11^ bladder cancer,^12^ melanoma,^13^ endometrial carcinoma,^14^ ovarian cancer,^15^ colorectal cancer 16 and gastric cancer.^17^ However, the involvement of miR‐612 in cervical cancer and its associated mechanism remains unclear.

NIN/RPN12 binding protein 1 (NOB1p), encoded by nin one binding protein (NOB1), has been revealed as an essential factor in 26S proteasome biogenesis that participates in protein degradation. High expression of NOB1 was observed during the carcinogenesis and progression of cervical cancer. MiRNAs have been shown to affect NOB1 expression in several cancers. For example, miR‐215 and miR‐363 targeted NOB1 and inhibited the growth and invasion of epithelial ovarian cancer cells, miR‐326 functioned as a tumour suppressor in glioma by targeting NOB1, and miR 744 suppressed the proliferation and invasion of papillary thyroid cancer cells by directly targeting NOB1. We speculated that NOB1 may function as an oncogene in cervical cancer and can be regulated by miRNAs.

In this work, we investigated the biological effect of miR‐612 on cervical cancer cell proliferation, apoptosis, migration and invasion in vitro and tumour growth in vivo. Moreover, we investigated the underlying mechanisms of NOB1 gene regulation by miR‐612 in cervical cancer.

## 2 MATERIALS AND METHODS

### 2.1 Tissue specimens

Human cervical cancer tissues and adjacent normal tissues were collected from 52 cervical cancer patients (range 36 to 77 years of age, median age 52.5) through surgery at the Second Hospital of Jilin University. Patients who received radiotherapy, chemotherapy or other anti‐cancer treatments before surgery were excluded. All samples were frozen in liquid nitrogen immediately after surgery and stored at −80°C. This work was approved by the Ethics Committee of the Second Hospital of Jilin University. Written informed consent to participate in this study was obtained from all patients.

### 2.2 Cell culture and transfection

Four types of human cervical cancer cells (SiHa, HeLa, C‐33‐A and Ca‐Ski) and the normal cervical epithelial cell line H8 were acquired from the American Type Culture Collection. The cells were maintained in Dulbecco's modified Eagle's medium (DMEM, Gibco) supplemented with 10% foetal bovine serum (FBS; Gibco), 100 U/mL penicillin (Gibco) and 100 mg/mL streptomycin (Gibco) at 37°C in a humidified atmosphere containing 5% CO_2_.

MiR‐612 mimics and corresponding negative controls (miR‐NC) were obtained from GenePharma Co. Ltd. NOB1 overexpression vectors (pCDNA3.1‐NOB1) were constructed and stored in our laboratory. SiHa cells were transfected with mimic, or plasmid vectors using Lipofectamine 2000 (Invitrogen) according to the manufacturer's procedures.

### 2.3 RNA extraction and quantitative reverse transcription‐polymerase chain reaction (qRT‐PCR)

Total RNA was extracted from tissues and cultured cells using TRIzol reagent (Invitrogen), followed by purification using an RNeasy Maxi kit (Qiagen). MiR‐612 expression was examined using the TaqMan microRNA Assay Kit (Thermo Fisher Scientific, Inc) in an ABI 7900 real‐time PCR system (Thermo Fisher Scientific, Inc) following the prescribed protocols. *NOB1* mRNA expression was detected as described in our previous study.^18^ The endogenous control for miR‐612 was U6 while that for *NOB1* was GAPDH. Relative expression levels were calculated by the 2^−ΔΔCt^ method using ABI software.^19^

### 2.4 Cell viability assay

Cell proliferation was detected by the Cell Counting Kit‐8 (CCK‐8) assay. Briefly, 5 × 10^3^ cells were seeded in 96‐well microtitre plates for 24 to 96 hours, and 10 μL of CCK‐8 reagent was added to each well on days 1, 2, 3 and 4. After 4 hours of culture at 37°C, the absorbance was recorded at 450 nm using a Benchmark Plus microplate spectrometer (Bio‐Rad Laboratories).

### 2.5 Cell apoptosis assay

The annexin V‐fluorescein isothiocyanate apoptosis detection kit (Sigma) and propidium iodide (Sigma) were utilized to determine cell apoptosis according to the manufacturer's protocols. The percentage of cell apoptosis was assessed by flow cytometry (FACScan, Becton‐Dickinson) following the instructions of the manufacturer.

### 2.6 Wound healing assay

The wound healing assay was performed to determine the migration ability. Growing transfected cells (1 × 105 cells/well) were seeded in six plates, and homogeneous wounds were formed in the cell monolayer with the tip of a sterile plastic micropipette. Images of wound closure were acquired at 0 and 24 hours using a Nikon Eclipse TS100 phase‐contrast microscope, and image analysis was carried out using Nikon NIS‐Element Basic Research v3.2 software.

### 2.7 Transwell invasion assay

The invasive capability of cervical cancer cells was assessed using an 8‐μm pore polycarbonate membrane Boyden chamber. The upper chambers were coated with Matrigel (BD) and seeded with 5 × 104 transfected cells in 200 μL of serum‐free DMEM, while 600 μL of media supplemented with 20% FBS was added to the lower chamber. After 24 hours, the invasive cells were fixed with 100% methanol for 30 minutes, after which the cells were stained using 0.1% crystal violet for 5 minutes. Five fields were randomly selected under an inverted optical microscope (Nikon) to evaluate the invasive ability of the cells by counting the number of invaded cells.

### 2.8 Bioinformatics analysis and luciferase reporter assay

Putative targets of miR‐612 were searched using TargetScan (http://targetscan.org/) and miRDB (http://www.mirdb.org/). NOB1, which was predicted as a target of miR‐612, was then assessed by luciferase reporter assay.

The 3'‐UTR of NOB1 containing either wild‐type (WT) or mutant‐type (MT) binding sites of miR‐612 were synthesized by GenePharma Co., Ltd. and inserted into the pmirGLO vector (Promega), with the resultant constructs denoted as WT‐NOB1 and MT‐NOB1, respectively. SiHa cells were cotransfected with miR‐612 mimics or miR‐NC and reporter plasmids WT‐NOB1 or MT‐NOB1 using Lipofectamine 2000. The activities of Renilla and firefly luciferase were examined using a Dual‐Luciferase^®^ Reporter assay kit from Promega based on the manufacturer's protocols. The activity of firefly luciferase was normalized to that of Renilla luciferase.

### 2.9 Western blot analyses

Western blot analyses was conducted as described in our previous work.^20^ Primary antibodies against NOB1 and GAPDH (control) and horseradish peroxidase‐linked secondary antibodies were purchased from Santa Cruz Biotechnology. The protein blots were detected using the SuperSignal West Pico Chemiluminescent Substrate kit (Pierce).

### 2.10 Xenograft tumour assay

All animal studies were performed in accordance with the guidelines of the Animal Care and Use Committee of Jilin University. Nude BALB/c mice (aged 4‐6 weeks; 18‐20 g) were obtained from the Jilin Laboratory Animal Center (Changchun, China) and housed in our laboratory under standard laboratory conditions. Cells (2 × 106) transfected with miR‐612 mimics or miR‐NC in 200 mL of DMEM were subcutaneously implanted into the left flanks of the animals (n = 5 per group). The width (W) and length (L) of the tumour xenografts were measured using a vernier calliper every five days, and the tumour volume was estimated as follows: volume = 0.5 × L × W^2^. On the 30th day, all mice were killed and the tumour xenografts were removed and weighed. A part of xenograft tissue was dissolved by RNA TRIzol lysate to further detect the expression of miR‐612 and NOB1 by qRT‐PCR.

### 2.11 Statistical analysis

The data are presented as the mean ± standard deviation of at least three replicates. All analysis was performed using SPSS v19.0 (IBM). Student's *t*‐tests were performed to compare the difference between two groups, and one‐way analysis of variance was carried out to compare the differences among more than two groups. The correlation between NOB1 and miR‐612 was assessed by Pearson's correlation analysis. *P* < .05 indicates statistical significance.

## 3 RESULTS

### 3.1 miR‐612 is down‐regulated in cervical cancer

To investigate the effect of miR‐612 on cervical cancer progression, we first detected the expression of miR‐612 in cervical cancer tissues and adjacent normal tissues by qRT‐PCR. We revealed that miR‐612 was significantly down‐regulated in cervical cancer samples relative to that in adjacent normal controls (Figure 1A). We next explored the relationship between miR‐612 and clinicopathological characteristics of cervical cancer patients. Based on the median value of miR‐612 expression (n = 52), the patients were separated into miR‐612‐low (n = 28) and miR‐612‐high (n = 24) groups. We found that miR‐612 expression was closely correlated with Fédération Internationale de Gynécologieetd'Obstétrique (FIGO) staging and lymph node metastasis (Table 1). We also examined miR‐612 expression in four types of human cervical cancer cells (SiHa, HeLa, C‐33‐A and Ca‐Ski) and normal cervical epithelial cells H8 by qRT‐PCR. Compared with H8 cells, all cervical cancer cell lines showed a lower expression of miR‐612 (Figure 1B). This finding indicates that miR‐612 may be a regulator of cervical cancer progression.

**Figure 1:** MiR‐612 is down‐regulated in cervical cancer tissues and cell lines. A, Relative miR‐612 expression levels in cervical cancer tissues and adjacent normal tissues were determined by qRT‐PCR. B, Expression of miR‐612 in four cervical cancer cell lines was significantly elevated relative to that in normal cervical epithelial cells H8. U6 was used as an internal control. **P < .01. Abbreviation: MiR, microRNA

**Table 1:** Correlation between clinicopathological features and miR‐612 expression in cervical cancer

Variables	No. of cases	miR‐612 expression		*P* value
		Low	High	
Age (years)				
<60	24	12	12	.7808
≥60	28	16	12	
HPV 16/18 infection				
Positive	32	20	12	.1556
Negative	20	8	12	
FIGO (Federation of Gynecology and Obstetrics staging system for cervical cancer) stage				
I‐II	38	15	23	.0006
III‐IV	14	13	1	
Tumour size				
<4	32	15	17	.2585
≥4	20	13	7	
Lymph node metastasis				
No	36	14	22	.0020
Yes	16	14	2	

### 3.2 miR‐612 inhibited cervical cancer cell proliferation and induced apoptosis

The biological activity of miR‐612 in the context of cervical cancer tumorigenesis was explored using SiHa cells transfected with miR‐612 mimics or miR‐NC, and the transfection efficiency was measured by qRT‐PCR. The results confirmed that after miR‐612 mimic transfection, the expression of miR‐612 was significantly elevated in SiHa cells relative to that in cells transfected with miR‐NC (Figure 2A). Subsequently, CCK‐8 assay was performed to assess the effect of miR‐612 on cell proliferation. We observed that miR‐612 overexpression significantly inhibited SiHa cell proliferation 48 to 96 hours after transfection (Figure 2B). Moreover, flow cytometry confirmed that miR‐612 mimic transfection promoted SiHa cell apoptosis to a greater extent relative to miR‐NC transfection (Figure 2C).

**Figure 2:** MiR‐612 inhibited cervical cancer cell proliferation and induced apoptosis. A, Relative miR‐612 expression levels in SiHa cells transfected with miR‐612 mimics or miR‐NC were measured by qRT‐PCR. B, The proliferation of SiHa cells transfected with miR‐612 mimics or miR‐NC was assessed by CCK‐8 assay. C, Apoptosis of SiHa cells transfected with miR‐612 mimics or miR‐NC was evaluated by flow cytometry. *P < .05; **P < .01. Abbreviations: CCK‐8, Cell Counting Kit‐8; MiR, microRNA; NC, negative control

### 3.3 miR‐612 inhibited cervical cancer cell migration and invasion

Next, we assessed the relationship between miR‐612 and cervical cancer cell migration and invasion using wound healing and Transwell invasion assays, respectively. SiHa cells transfected with miR‐612 showed significantly reduced cell migration and invasion compared to those of miR‐NC‐transfected cells (Figure 3A,B).

**Figure 3:** MiR‐612 inhibited cervical cancer cell migration and invasion. A, Migration of SiHa cells transfected with miR‐612 mimics or miR‐NC was examined by wound healing assay. B, Invasion of SiHa cells transfected with miR‐612 mimics or miR‐NC was assessed by the Transwell invasion assay. **P < .01. Abbreviations: MiR, microRNA; NC, negative control

### 3.4 NOB1 is a target of miR‐612 in cervical cancer cells

Bioinformatics prediction revealed potential binding sites of miR‐612 on the 3'‐UTR of NOB1 (Figure 4A). A luciferase reporter assay was conducted in SiHa cells to confirm this finding. miR‐612 overexpression significantly lowered luciferase activity in WT‐NOB1 but had no effect on MT‐NOB1 (Figure 4B). Moreover, miR‐612 overexpression significantly reduced the protein and mRNA expression of NOB1 (Figure 4C,D). We also observed that NOB1 levels were elevated in cervical cancer tissues compared to that in adjacent normal control samples (Figure 4E). In addition, a negative correlation between miR‐612 and NOB1 was revealed in cervical cancer tissues (*r* = −.631, *P* < .001; Figure 4F). These findings collectively indicate that NOB1 is a target of miR‐612 in cervical cancer cells.

**Figure 4:** NOB1 is a direct target of miR‐612 in cervical cancer cells. A, MiR‐612 and its putative binding sequence and mutated binding sites in the NOB1 3′‐UTR. B, MiR‐612 overexpression significantly suppressed the luciferase activity of WT‐NOB1, but not MT‐NOB1. (C, D) mRNA and protein expression of NOB1 in SiHa cells transfected with miR‐612 mimics or miR‐NC were determined by qRT‐PCR and Western blot analyses, respectively. GAPDH was used as an internal control. E, *NOB1* mRNA expression was detected in cervical cancer tissues and adjacent normal tissues. F, A significant inverse correlation between the *NOB1* mRNA levels and miR‐612 was observed in cervical cancer tissues. **P < .01. Abbreviations: MiR, microRNA; MUT, mutated; NC, negative control; NOB1, nin one binding protein; UTR, untranslated region; WT, wild‐type

### 3.5 Overexpression of NOB1 rescued cervical cancer cells from miR‐612‐mediated anti‐cancer activity

To assess the extent to which miR‐612 regulates NOB1, we conducted rescue experiments by transfecting miR‐612‐overexpressing SiHa cells with NOB1 overexpression (pCDNA3.1‐NOB1) plasmids. We found that transfection of pCDNA3.1‐NOB1 in SiHa cells restored NOB1 expression, which in turn led to a reduction in miR‐612 expression (Figure 5A,B). Furthermore, restoration of SOX12 partially counteracted the effects of miR‐612 overexpression on SiHa cells in terms of proliferation, apoptosis, migration and invasion (Figure 5C‐F).

**Figure 5:** NOB1 overexpression partially counteracted miR‐612‐mediated decrease in cervical cancer cell proliferation, migration and invasion. (A, B) mRNA and protein expression of NOB1 in SiHa cells after transfection with miR‐612 mimics with (or without) NOB1 overexpression (pCDNA3.1‐NOB1) vector or miR‐NC. GAPDH was used as an internal control. (C–F) Cell proliferation, apoptosis, migration and invasion were evaluated in SiHa cells after transfection with miR‐612 mimics with (or without) pCDNA3.1‐NOB1 or miR‐NC. *P < .05; **P < .01. Abbreviations: miR, microRNA; NC, negative control; NOB1, nin one binding protein

### 3.6 miR‐612 suppressed tumour growth in vivo

SiHa cells transfected using either miR‐612 mimics or miR‐NC were implanted into nude mice to study the effect of miR‐612 on tumour growth in vivo. We evaluated the tumours every 5 days after implantation and found that miR‐612 mimics induced notably slower tumour growth than did miR‐NC (Figure 6A, *P* < .05). The experimental mice were killed 30 days after implantation, at which time the tumours were excised and weighed. We observed that tumour weight and size were notably decreased in the miR‐612 group compared to those in the miR‐NC group (Figure 6B,C). Moreover, we examined the expression of miR‐612 and NOB1 in the xenografted tumours and revealed that miR‐612 was down‐regulated, whereas NOB1 was up‐regulated in the tumour tissues of the miR‐612 group (Figure 6D).

**Figure 6:** MiR‐612 suppressed tumour growth in vivo. A, Tumour volume was measured every five days until mice were killed. B, Images of the xenografted tumour. C, Weight of the xenografted tumour. D, Relative expression of miR‐612 and NOB1 in xenografts was determined by qRT‐PCR. *P < .05; **P < .01. Abbreviations: miR, microRNA; NC, negative control; NOB1, nin one binding protein

## 4 DISCUSSION

miRNA dysregulation plays a crucial role in the occurrence and progression of cervical cancer via the regulation of cancer cell proliferation, migration, invasion and metastasis.^9^, ^10^ Further studies on the regulatory function of miRNAs and their potential molecular mechanisms in cervical cancer may aid in identifying diagnostic markers and therapeutic targets. MiR‐612 has been shown to exhibit tumour‐suppressing activity in multiple cancers by regulating major tumour‐related biological behaviours.^11^, ^12^, ^13^, ^14^, ^15^, ^16^, ^17^ However, the expression status and associated mechanisms of miR‐612 in cervical cancer remain unclear. Here, we detected miR‐612 expression in cervical cancer samples and determined the clinical significance of this tumour. Additionally, we explored the role and underlying mechanisms of miR‐612 in cervical cancer. We found that miR‐612 levels were decreased in cervical cancer tissues and cell lines were linked to the FIGO stage and lymph node metastasis. In addition, miR‐612 inhibited cervical cancer growth by regulating NOB1. Functional experiments revealed that miR‐612 overexpression restricted the proliferation, induced the apoptosis, and inhibited the migration and invasion of these cancer cells in vitro, while also suppressing in vivo tumour growth. This indicates that miR‐612 may be a potential biomarker or therapeutic target of cervical cancer.

MiRNAs are generally known to alter biological processes by regulating target genes.^4^, ^6^ To investigate how miR‐612 inhibits cervical cancer, its potential targets were identified by bioinformatics analysis. Among the targets, NOB1 was chosen as a subject of study based on its biological function.^21^, ^22^

NOB1 was reportedly linked to the onset and development of various tumours and plays the role of an oncogene.^23^, ^24^, ^25^, ^26^, ^27^ A previous study showed that NOB1 levels were elevated in cervical cancer tissues and cell lines.^28^ Studies have also demonstrated that miR‐139‐3p inhibited cervical cancer cell proliferation, migration, and invasion and induced cell apoptosis through down‐regulation of NOB1 expression. In line with this result, we further confirmed that NOB1 expression was up‐regulated in cervical cancer tissues relative to that in adjacent normal tissues. We confirmed that NOB1 was a target of miR‐612 in cervical cancer using luciferase reporter assay, Western blot analyses and qRT‐PCR. Moreover, NOB1 overexpression partially blocked the effect of miR‐612 on cervical cancer cell proliferation, apoptosis, migration and invasion. These data provided reliable evidence that miR‐612 inhibits cervical cancer progression, at least to some extent, by inhibiting the expression of NOB1.

## 5 CONCLUSION

Herein, we found that miR‐612 expression was decreased in cervical cancer tissues and cell lines and was related to lymph node metastasis. Our data indicated that miR‐612 targeted NOB1 to inhibit cervical cancer cell proliferation, migration and invasion and induce apoptosis in vitro, while also suppressing tumour growth in vivo. The findings indicate that miR‐612 may be a potential therapeutic target for cervical cancer treatment.

## CONFLICT OF INTEREST

The authors confirm that there are no conflicts of interest.

## AUTHOR CONTRIBUTION

YL contributed to the conception and design of the study; YJ, XXY and ZZ performed the statistical analysis and prepared the first draft of the manuscript; XZ wrote sections of the manuscript; MC provided critical revisions. All authors contributed to manuscript revision and have read and approved the submitted version.

## Data Availability

Research data are not shared.
